# Asymmetric white matter degeneration in amyotrophic lateral sclerosis: a diffusion kurtosis imaging study of motor and extra-motor pathways

**DOI:** 10.3389/fnins.2025.1581719

**Published:** 2025-04-25

**Authors:** Juan Carlos Quizhpilema, Ane Legarda, José Manuel Hidalgo, Pablo Lecumberri, Ivonne Jerico, Teresa Cabada

**Affiliations:** ^1^Universidad Publica de Navarra, Department of Statistics, Computer Science and Mathematics, Pamplona, Spain; ^2^Department of Radiology, Hospital Universitario de Navarra (HUN), Pamplona, Spain; ^3^Department of Neurology, Hospital Universitario de Navarra (HUN), Pamplona, Spain; ^4^IdiSNA, Navarra Institute for Health Research, Pamplona, Spain

**Keywords:** amyotrophic lateral sclerosis, diffusion kurtosis imaging, white matter, tractography, biomarkers, corticospinal tract, neurodegeneration, diffusion MRI

## Abstract

**Background:**

Amyotrophic Lateral Sclerosis (ALS) is a progressive neurodegenerative disease that lacks effective early biomarkers. This study investigated the potential of diffusion kurtosis imaging (DKI) as a non-invasive biomarker for detecting and monitoring ALS progression through a comprehensive analysis of white matter alterations.

**Methods:**

We performed a cross-sectional analysis of magnetic resonance images with advanced diffusion imaging techniques in ALS patients recruited from a neurodegenerative consultation service over a 3-year period and healthy controls. Our methodology employed multi-shell multi-tissue constrained spherical deconvolution (MSMT-CSD) for tract reconstruction and diffusion kurtosis imaging for microstructural analysis. The study focused particularly on the corticospinal tract and associated pathways, utilizing both tract-specific Bundle Analytics (BUAN) and whole-brain Tract-Based Spatial Statistics (TBSS) approaches.

**Results:**

The study included 33 ALS patients and 37 controls with no significant differences in age or gender. ALS patients predominantly presented with spinal onset and exhibited moderate functional impairment (ALSFRS-R: 39.09 ± 5). Whole-brain TBSS revealed widespread white matter alterations, with increased MD, RD, and AD, and decreased FA notably in the corona radiata, internal capsule, and corticospinal tracts. Detailed fiber tracking of the corticospinal tracts showed significant microstructural changes, with the left CST displaying pronounced increases in MD and AD alongside reduced FA, while the right CST exhibited distinctive regional variations. Additionally, analyses of the frontopontine and parietopontine tracts uncovered further alterations in diffusion metrics. Despite imaging findings, clinical-radiological correlations with functional scores and disease progression were not statistically significant.

**Conclusions:**

This study explores DKI as a potential biomarker for ALS pathology, revealing microstructural changes in both motor and extra-motor pathways. Using whole-brain TBSS analysis and tractography with DIPY, we identified an asymmetric pattern of degeneration and involvement of integrative neural networks, providing new insights into ALS pathophysiology. These findings contribute to our understanding of the complex structural alterations in ALS and suggest that DKI-derived metrics may have utility in characterizing the disease process.

## 1 Introduction

Amyotrophic Lateral Sclerosis (ALS) is a fatal neurodegenerative disorder characterized by progressive degeneration of upper motor neurons (UMN) and lower motor neurons (LMN), with a median survival of 2–5 years post-diagnosis (Brown and Al-Chalabi, 2017). Despite advances in molecular characterization, early diagnosis remains hampered by clinical heterogeneity and the absence of biomarkers detecting pre-symptomatic axonal degeneration (Goutman et al., 2022). The diagnosis of ALS remains primarily clinical, following a complex process that often results in significant diagnostic delays. The current diagnostic framework relies on the revised El Escorial criteria (Brooks et al., 2000), which were updated in 2015 (Ludolph et al., 2015) to improve diagnostic sensitivity while maintaining specificity. However, several challenges persist in the early and accurate diagnosis of ALS.

Early symptoms can be subtle and non-specific, often resembling other neurological conditions. Physical examination focuses on identifying both upper motor neuron and lower motor neuron signs, but the heterogeneous presentation of these signs can complicate early diagnosis. Progressive muscle weakness typically begins focally, making it challenging to differentiate from other neuromuscular conditions (Hardiman et al., 2017).

Electrophysiological (EMG) studies and nerve conduction studies (NCS) have been essential diagnostic tools, but these techniques have limits in detecting early changes in denervation. These techniques do not allow detection of abnormalities until there is a significant loss of motor neurons, requiring about 30% motor neuron loss (Lari et al., 2019). Furthermore, EMG findings can be non-specific and may appear similar to other neuromuscular disorders.

Current biomarkers lack sufficient sensitivity and specificity for early diagnosis. Neurofilament light chain (NfL) levels in cerebrospinal fluid and blood show promise but are not yet validated for routine clinical use. The absence of a definitive biomarker significantly impacts early diagnosis and disease monitoring (Poesen et al., 2017).

Conventional magnetic resonance imaging (MRI) is primarily used to exclude other conditions rather than confirm ALS diagnosis. While advanced neuroimaging techniques show promise in detecting early neural pathway changes, they are not yet part of standard diagnostic criteria (Turner et al., 2009). However, the active search for biomarkers for the detection of the disease does not cease, different investigations carried out in the field of MRI have provided a lot of information.

Advanced neuroimaging techniques have emerged as promising tools for the detection and monitoring of ALS, offering insights beyond conventional MRI.

Diffusion tensor imaging (DTI) has emerged as a particularly valuable technique for investigating microstructural alterations in ALS, with meta-analyses confirming consistent abnormalities in white matter tracts, especially the corticospinal tract (Li et al., 2012; Foerster et al., 2013). Despite its widespread application, the diagnostic utility of DTI metrics has been limited by methodological heterogeneity and the complex pathophysiology of ALS, necessitating careful interpretation of imaging findings (Bede and Hardiman, 2014). Recent studies have demonstrated the potential of DTI parameters as biomarkers for ALS, showing significant correlations with clinical measures and disease progression (Baek et al., 2020). However, the sensitivity and specificity of single-modality approaches remain suboptimal for individual patient assessment. To address these limitations, multimodal MRI approaches that integrate structural, diffusion, and functional techniques have shown promising results, improving diagnostic accuracy and sensitivity to longitudinal changes in ALS (Pisharady et al., 2023).

Studies, where diffusion tensor imaging (DTI) has been applied, have shown significant alterations in fractional anisotropy (FA) and mean diffusivity (MD) values in ALS patients compared to healthy controls, and these changes correlate with disease progression and functional impairment (Chió et al., 2014). Nevertheless, DTI techniques have limitations to reliance on Gaussian diffusion models, which oversimplify the complex microstructure of degenerating white matter (Assaf and Pasternak, 2008). Diffusion kurtosis imaging (DKI) addresses these limitations by quantifying non-Gaussian water diffusion, revealing microstructural features such as axonal density, dendritic complexity, and glial reactivity–key pathological hallmarks in ALS (Jensen and Helpern, 2010).

DKI captures non-Gaussian water diffusion properties, offering more detailed information about tissue complexity and cellular barriers than conventional DTI. Studies implementing DKI have revealed significant alterations in mean kurtosis (MK) values in the motor cortex and along the CST of ALS patients, potentially serving as earlier and more sensitive markers of neurodegeneration (Andica et al., 2020; Chen et al., 2017). These findings suggest that DKI metrics might detect pathological changes even before conventional DTI parameters show significant alterations (Welton et al., 2019). However, inconsistencies in analytical approaches and limited focus on extramotor pathways hinder clinical translation (Bede and Hardiman, 2018).

Recent developments in fiber tractography, combining both DTI and DKI approaches, have enabled more comprehensive mapping of white matter pathway alterations in ALS. These advanced tractography methods have revealed specific patterns of degeneration along the CST, with changes often beginning in the primary motor cortex and progressing causally, offering new perspectives on the pathophysiological mechanisms underlying ALS progression (Anand et al., 2023).

Despite advances in neuroimaging techniques, there remains a critical need for sensitive and reliable biomarkers that can detect early microstructural changes in amyotrophic lateral sclerosis. While diffusion tensor imaging has shown promise in identifying white matter alterations, its inability to capture non-Gaussian water diffusion potentially limits its sensitivity to complex tissue changes (Steven et al., 2014). Our research proposes that DKI assessment within sensorimotor tracts will reveal distinct patterns of microstructural degeneration in ALS patients, with metrics that correlate significantly with clinical measures of upper motor neuron dysfunction and disease progression. The application of DKI metrics is expected to demonstrate superior sensitivity in detecting pathological changes compared to conventional diffusion tensor parameters, especially in regions where traditional measures remain within normal ranges (Steven et al., 2014). Moreover, the integration of advanced 3D fiber tractography techniques will provide unprecedented visualization of these microstructural alterations, offering a comprehensive spatial mapping of disease-related pathology along these critical white matter pathways. This multi-modal approach aims to establish DKI as a robust biomarker for detecting microstructural alterations in ALS patients, potentially advancing our understanding of the disease's underlying pathophysiology at the time of diagnosis.

## 2 Methods

### 2.1 Participants

The recruitment of ALS cases and controls was carried out in the ALS unit of the University Hospital of Navarra (HUN) for three consecutive years.

The inclusion criteria for the patient group was a diagnosis of probable or defined ALS according to the El Escorial criteria. Patients were excluded if they had a medical history of cerebral ischemic events, other previous neurodegenerative or neuropsychiatric diseases, significant respiratory insufficiency, or contraindications for MRI. In the healthy control group, subjects had no family history of neurodegenerative disease, no history of severe head trauma, ischemic events, or any other serious neurological, psychiatric, or other diseases.

This study was reviewed and approved by the local ethics committee, and written informed consent was obtained from all participants.

### 2.2 Data acquisition

The MRI studies were carried out on a 3T MAGNETON Vida system (Siemens Healthineers, Erlangen, Germany) using a 32-channel head coil array, with the following imaging parameters for each technique:

High-resolution T1-weighted structural images were acquired using a three-dimensional magnetization-prepared rapid gradient-echo (MPRAGE) sequence with inversion time (TI) = 1,020 ms, echo time (TE) = 2.61 ms, repetition time (TR) = 2,100 ms, field of view (FoV) = 230 × 230 mm^2^, acquisition matrix = 256 × 256, and 192 sagittal slices. The sequence employed a GRAPPA acceleration factor of 3, yielding an isotropic voxel resolution of 0.9 mm^3^.

The diffusion weighting data were acquired using a multi-shell acquisition protocol with 64 diffusion-encoding directions. The protocol included three b-values (b = 0, 1,000, and 2,000 s/mm^2^) to enable advanced diffusion modeling, resulting in a total of 140 diffusion-weighted volumes, each containing 66 anatomical slices. The sequence parameters were: echo time (TE) = 91 ms, repetition time (TR) = 3,800 ms, with a field of view (FoV) = 200 × 200 mm^2^, and acquisition matrix = 100 × 100. The protocol employed a simultaneous multi-slice (SMS) acceleration factor of 3 and GRAPPA parallel imaging acceleration factor of 2, resulting in an isotropic voxel resolution of 2 mm^3^.

Clinical and neurophysiological data were obtained concurrently with MRI acquisition. Functional status was evaluated using the Amyotrophic Lateral Sclerosis Functional Rating Scale-Revised (ALSFRS-R) and disease progression rate was calculated as (48 - ALSFRS-R score)/symptom duration in months.

### 2.3 MRI analysis

#### 2.3.1 Data preprocessing

The diffusion-weighted and T1-weighted images were visually inspected for possible acquisition problems such as motion, susceptibility, and artifact noise. As a first step, all acquisitions were subjected to an initial pre-processing to correct acquisition problems.

All raw diffusion scans were denoised using the Diffusion Imaging in Python (DIPY https://dipy.org/index.html) (Garyfallidis et al., 2014) software package applying self-supervised denoising via statistical independence (Fadnavis et al., 2020) and motion corrected (Jenkinson and Smith, 2001). Distortion susceptibility was corrected using topup (Andersson et al., 2003) of FSL's (Jenkinson et al., 2012). Before performing the susceptibility correction, Synb0-DiscCO (Schilling et al., 2020) was used to synthesize a distortion-free image b = 0. Eddy current correction is performed using eddy (Andersson and Sotiropoulos, 2016) of FSL implementation, the b matrix was rotated to preserve the correct orientation information after the eddy current and tilt angle corrections (Leemans and Jones, 2009). Finally, a Gibbs ring correction is applied to reduce artifacts in the white matter (Veraart et al., 2016). Additionally, the T1-weighted images were denoised using the Non-Local Means (Coupe et al., 2008).

All diffusion image processing, including both the reconstruction of diffusion models and fiber tracking procedures, was performed using the DIPY software package (version 1.9.0), a comprehensive library for diffusion MRI analysis and tractography.

#### 2.3.2 DWI reconstruction

Diffusion reconstruction was performed using two complementary models. First, DKI (Jensen and Helpern, 2010; Henriques et al., 2021) was implemented to obtain enhanced diffusion metrics, including fractional anisotropy (FA), mean diffusivity (MD), axial diffusivity (AD), and radial diffusivity (RD). Subsequently, Multi-Shell Multi-Tissue Constrained Spherical Deconvolution (MSMT-CSD) (Jeurissen et al., 2014) was applied to optimize tractographic reconstruction, allowing a more accurate characterization of tract anatomy.

Prior to diffusion metric computation, a binary mask was applied to the diffusion-weighted images to exclude background noise and non-brain tissue. The DKI model was then fitted to the masked diffusion data to estimate multiple diffusion metrics: FA, AD, MD, and RD. These metrics were computed for each voxel within the brain mask to quantify local water diffusion properties.

For the reconstruction of fiber orientations, T1-weighted images were first used to perform tissue segmentation, distinguishing between white matter, gray matter, and cerebrospinal fluid. These tissue maps were then incorporated into the Multi-Shell Multi-Tissue Constrained Spherical Deconvolution (MSMT-CSD) method. This technique takes advantage of both the tissue segmentation and the additional information provided by different b-values to separate the contributions from different tissues and provide a more accurate estimation of fiber orientations. The response function for each tissue was estimated in a tissue-specific manner using an iterative self-calibration process adapted for multi-shell data.

#### 2.3.3 DWI fiber traking

The fiber tracking of white matter was performed using the parallel transport algorithm (Aydogan and Shi, 2021), which preserves the local differential geometry of diffusion space. To ensure anatomical specificity, the tractography was constrained using tissue-specific masks derived directly from MSMT-CSD analysis and T1 segmentation.

For quantitative analysis of the reconstructed tracts, scalar metrics were mapped onto each streamline using DIPY. This process involved interpolating the scalar values from the DKI metric maps at each point along the streamlines, allowing for detailed characterization of microstructural properties along the entire length of each tract. The mapping was performed using a trilinear interpolation method to ensure accurate sampling of the scalar values while maintaining the native resolution of the diffusion data.

#### 2.3.4 Tract segmentation analysis

In our tract segmentation analysis, each reconstructed white matter tract is divided into 100 segments through the creation of assignment maps in a common model space. This approach, as described in previous studies (Garyfallidis et al., 2012, 2014), allows us to capture local variations in diffusion properties—such as fractional anisotropy (FA)—that might be overlooked when the entire tract is analyzed as a single entity. By assigning each point on a streamline to its nearest segment based on Euclidean distance, we preserve the natural distribution of points without re-sampling, ensuring that regional differences in tract integrity are accurately reflected.

#### 2.3.5 TBSS

Following the initial preprocessing steps and diffusion metric computation described above, the data were further analyzed using Tract-Based Spatial Statistics (TBSS) (Smith et al., 2006). Using the previously obtained diffusion metrics (FA, MD, AD, and RD) derived from the DKI model, all subjects' FA images were nonlinearly registered to a common space. Next, a mean FA image was created and thinned to generate a mean FA skeleton, which represents the centers of all white matter tracts common to the group. This skeleton was thresholded at *FA*>0.2 to exclude peripheral tracts with high inter-subject variability and partial volume effects. Subsequently, each subject's aligned FA data was projected onto this skeleton for voxelwise cross-subject statistical analysis. The transformation matrices derived from the FA images were then applied to the other diffusion metrics (MD, AD, and RD) to allow for multi-metric voxelwise statistical analysis.

### 2.4 Statistical analysis

Demographic comparisons between ALS patients and healthy controls were conducted using appropriate statistical tests. Age differences were assessed using two-sample independent t-tests, while gender distribution was analyzed using chi-squared test. For the ALS group, clinical characteristics including disease duration, ALSFRS-R scores, and progression rates were summarized using descriptive statistics.

Neuroimaging analyses were performed using two complementary methodological approaches to comprehensively assess white matter alterations.

The first approach is whole brain analysis, voxelwise statistical tests were performed using FSL's randomize tool, implementing nonparametric permutation tests with 500 permutations. The analysis included age and sex as covariates to control for demographic effects. Correction for multiple comparisons was performed using threshold-free cluster enhancement (TFCE), and statistical significance was set at *p* < 0.05 corrected. This dual analytic approach allowed both detailed examination of specific tracts of interest and comprehensive assessment of whole-brain white matter changes.

The second approach consists of an analysis using the Bundle Analytics (BUAN) module within DIPY to examine tract-specific changes. Linear mixed models (LMM) were implemented to analyze differences in diffusion metrics along the corticospinal tract and associated white matter pathways. The statistical model incorporated group status as the main factor of interest while controlling for age, sex, and ALSFRS-R scores as covariates. Subject-specific random effects were included to account for individual variability in tract measurements. Statistical significance was assessed using a hierarchical approach with multiple thresholds (*p* < 0.05 and *p* < 0.01) to control for multiple comparisons across tract profiles.

Correlation analyses examined the relationships between diffusion metrics and clinical variables. Pearson's correlation coefficients were calculated to assess the associations between the average value of diffusion parameters (FA, MD, AD, and RD) along fiber tracts and clinical measures, specifically the ALSFRS-R scores and disease progression rate. Statistical significance was set at *p* < 0.05.

## 3 Results

### 3.1 Demographic and clinical characteristics

The study included 33 ALS patients (19 males, 14 females) and 37 controls (16 males, 21 females), with no significant differences in age (64.6 ± 10.35 vs. 60.8 ± 9.7 years, *p* = 0.114) or gender distribution (*p* = 0.144) (Table 1).

**Table 1:** Comparison between patients and controls.

**Characteristics**	**Controls**	**Patients**	***p*-Values**
n	37	33	
Age, years	60.8 ± 9.7	64.6 ± 10.35	0.114^a^
Gender (male, female)	16, 21	19, 14	0.144^b^

^a^Two-sample independent *t*-test.

^b^Chi-squared test.

Among ALS patients, the distribution of symptom onset patterns was spinal onset being predominant (66.7%, *n* = 22), followed by bulbar onset (27.3%, *n* = 9), and a small proportion presenting with generalized onset (6.0%, *n* = 2) (Table 2). The analysis of disease characteristics revealed that patients had a mean symptom duration of 27.46 ± 20.40 months at the time of MRI acquisition (Table 2). Laterality of initial symptoms show no significant differences in distribution (*p* = 0.307). Functional status assessment indicated moderate impairment, with a mean ALSFRS-R score of 39.09 ± 5 out of 48, and a disease progression rate of 0.38 ± 0.38. One patient was excluded from the ALSFRS-R analysis due to missing data (Table 2).

**Table 2:** Clinical characteristics of ALS patients.

**Characteristics**	**Values**	***p*-Values**
Symptom onset [n, (%)]		
Bulbar	9 (27.3)	
Spinal	22 (66.7)	
Generalized	2 (6.0)	
Symptom duration before MRI (months)	27.46 ± 20.40	-
ALSFRS-R/48 score	39.09 ± 5^b^	-
Disease progression rate	0.38 ± 0.38^b^	-
Initial symptoms of laterality [n, (%)]		0.307^a^
Left	10 (30.3)	
Right	8 (24.2)	
Others	15 (45.5)	

ALSFRS-R, Amyotrophic Lateral Sclerosis Functional Rating Scale-Revised.

^a^Chi-squared test.

^b^One patient was excluded because of missing ALSFRS-R score.

### 3.2 Whole-brain white matter analysis

Tract-Based Spatial Statistics (TBSS) analysis revealed significant white matter alterations in all diffusion metrics with a left predominance (Figure 1). We corrected for multiple comparisons using TFCE and *p* < 0.05 for the MD, RD, and AD metrics and *p* < 0.05 uncorrected for the FA diffusion metric.

**Figure 1:** Voxel-wise comparison of diffusion metrics (MD, FA, RD, and AD) displayed on axial brain slices (z = –32 to 68 mm). Green outlines show a white matter skeleton. Blue regions indicate areas where *patients*>*controls*, while brown/red regions (in FA) show areas where *patients*<*controls*. Images in radiological convention (R: Right, L: Left).

Multiple comparison correction was not applied to the FA analyses because the effects on FA were more subtle than on the other diffusion metrics. When applying multiple comparison correction to FA, an insufficient number of voxels exceeded the threshold to allow meaningful interpretation of corticospinal tract alterations. Uncorrected FA results are presented as exploratory findings.

MD showed increased bilateral diffusivity (z = 28–68), predominantly affecting the corona radiata and internal capsule. FA showed markedly decreased values (shown in red/brown) in the anterior and superior regions of the white matter, with marked involvement of the corticospinal tract. RD showed a pronounced increase in diffusivity (shown in blue) concentrated in the central areas of the white matter, from the corona radiata to the internal capsule. In addition, AD showed increased diffusivity along the white matter tracts. The most significant changes for MD, FA, and RD were observed in anterior and superior brain regions (z = 18–48).

### 3.3 Alterations of the corticospinal tract in fiber tracking

The corticospinal tract, being the principal motor pathway and a known site of pathology in ALS, demonstrated the most pronounced changes in our analysis. As shown (Figure 2), both left and right CST showed altered DKI parameters along their trajectories, with significant differences (*p* < 0.05).

**Figure 2:** Analysis of bilateral CST in ALS patients vs. controls, showing **(a)** left MD, **(b)** right MD, **(c)** left FA, **(d)** right FA, **(e)** left RD, **(f)** right RD, **(g)** left AD and **(h)** right RD, for both groups along tract segments (0–100). Blue bars represent the p-value of the two-sample test, with blue and red thresholds indicating statistical significance (*p* < 0.05 and *p* < 0.01).

#### 3.3.1 Left corticospinal tract

Analysis of the left corticospinal tract revealed significant microstructural alterations in multiple diffusion metrics (Figure 3). MD values showed higher mean values in patients (red line) compared to controls (green line), with statistically significant differences particularly evident at segments 50–90 (*p* < 0.05) and more pronounced differences at segments 70–75, 85–90 (*p* < 0.01). FA trajectories showed maximum values around segments 35–45, where both groups reached peaks between 0.75–0.80, and patients exhibited lower mean values and significant reductions compared to controls at segments 35–40 (*p* < 0.05). FA differences became most evident in segments 90–95, where the patient group consistently showed reduced values. RD analysis revealed similar trajectory patterns between groups with initially elevated peaks at segments 0–5, followed by similar trajectories between segments. A notable separation occurred at segments 35–40 and 80–95, where patients showed elevated mean values compared to controls, with multiple segments reaching statistical significance thresholds (*p* < 0.05). AD demonstrated significantly higher patient values at segments 55–85 (*p* < 0.05), and particularly prominent differences at segments 65–85 (*p* < 0.01). The AD trajectory showed a characteristic pattern with elevated values in the middle portions (segments 20–60), reaching peaks of approximately 0.00175 mm^2^/s in the patient group, before gradually decreasing toward the tract endpoints.

**Figure 3:** 3D representation of the statistical significance (*p*>0.05) of the **(a)** MD, **(b)** FA, **(c)** RD, and **(d)** AD over the left CST tract. Red stripe significant values, blue stripe non-significant values.

#### 3.3.2 Right corticospinal tract

The right corticospinal tract exhibited a pattern of changes that revealed distinctive microstructural alterations in multiple diffusion metrics (Figure 4). MD values in patients (red line) showed similar trajectories to controls (green line) with subtle variations, particularly in segments 70–100 where patients showed slightly elevated values, although statistical significance was not achieved (*p* < 0.05). FA demonstrated maximal values in segments 35–45, reaching peaks of approximately 0.70–0.75, with patients showing consistently lower mean values. Notable reductions in FA were observed in segments 30–35 (*p* < 0.01), primarily affecting the central region of the tract. RD analysis showed an initial peak in segments 0–5, followed by stable trajectories in both groups. The patient group showed slightly elevated RD values throughout the tract length, with scattered segments reaching statistical significance (*p* < 0.05), particularly at segments 5–10 and 85–90. AD values showed the most prominent differences between groups, with controls showing higher mean values, particularly at segments 25–40, where peak values reached approximately 0.00175 mm^2^/s and patients showing slightly lower values, and notable differences at segments 80–90, although most differences remained at significance level *p* < 0.05. The AD trajectory showed a characteristic pattern with elevated values in the middle portions (segments 25–50) before gradually decreasing toward the endpoints of the tract reaching significance at segments 30–40 and 75–80 at *p* < 0.05. These findings were visualized in three-dimensional reconstructions, with color-coded representations highlighting the spatial distribution of these alterations along the length of the tract. This pattern of changes, although similar to that observed in the left corticospinal tract, showed a distinctive regional involvement.

**Figure 4:** 3D representation of the statistical significance (*p*>0.05) of the **(a)** MD, **(b)** FA, **(c)** RD, and **(d)** AD over the right CST tract. Red stripe significant values, blue stripe non-significant values.

Analysis of the aforementioned corticospinal tracts revealed differences in diffusion metrics between ALS patients and controls. The pattern of changes suggests a possible superior-to-inferior gradient of pathological involvement, which may reflect the progressive nature of ALS. Moreover, the alterations showed distinct patterns of involvement between the left and right hemispheres, suggesting potential asymmetric progression of pathology in ALS, a finding that may have important implications for understanding disease progression.

### 3.4 Extended white matter pathway involvement

Our analysis revealed that white matter alterations in ALS extend beyond the primary motor pathways, affecting several associated tracts crucial for motor function and cognitive processing. This broader involvement may help explain the spectrum of clinical manifestations observed in ALS patients.

#### 3.4.1 Frontopontine tract

Analysis of the left frontopontine tract revealed distinctive patterns of microstructural alterations (Figure 5). In the left tract, MD demonstrated significant differences at segments 60–85 (*p* < 0.05) with two segments reaching statistical significance (*p* < 0.01). FA reached maximal values of approximately 0.70–0.75 at segments 30–45, and patients showed subtle reductions throughout the tract reaching statistical significance at segments 5–10, 30–35, and 95–100 (*p* < 0.05). RD exhibited consistent elevations in patients across all segments reaching statistical significance at segments 30–35 and 85–90 (*p* < 0.05). AD values showed markedly elevated trajectories in patients compared to controls, particularly in segments 60-85 (*p* < 0.05), with peak values reaching approximately 0.00175 mm^2^/s in segments 20–25, Figure 5 shows the projection in the reconstructed 3D tracts.

**Figure 5:** Analysis of left FPT in ALS patients vs. controls, showing **(a)** MD and **(b)** FA for both groups across tract segments (0–100). Blue bars represent the *p*-value of the two-sample test, with blue and red thresholds indicating statistical significance (*p* < 0.05 and *p* < 0.01). This is complemented by a 3D representation of the left FPT tract showing in red the segments where there are significant differences between groups (*p* < 0.05) no significant differences were found on the right side.

#### 3.4.2 Parietopontine tract

Analysis of left parietopontine tracts revealed distinct patterns of microstructural changes (Figure 6). In the left tract, MD measures demonstrated increased values in patients, particularly between segments 60–85 (*p* < 0.05). FA showed maximum values around segments 35–45 (approximately 0.75–0.80), with patients showing subtle reductions throughout reaching statistical significance at segments 0–5, 85–100 (*p* < 0.05). AD values showed markedly elevated trajectories in patients compared to controls at segments 20–40 (peaking at approximately 0.00165 mm^2^/s) and maintained higher values at segments 60–80, with consistent statistical significance (*p* < 0.05), Figure 6 shows the projection in the reconstructed 3D tracts.

**Figure 6:** Analysis of left PPT in ALS patients vs. controls, showing **(a)** MD and **(b)** FA for both groups across tract segments (0–100). Blue bars represent the *p*-value of the two-sample test, with blue and red thresholds indicating statistical significance (*p* < 0.05 and *p* < 0.01). This is complemented by a 3D representation of the left PPT tract showing in red the segments where there are significant differences between groups (*p* < 0.05) no significant differences were found on the right side.

### 3.5 Clinical-radiological correlations

Correlations between diffusivity metrics (MD, FA, RD, and AD) and the clinical parameters evaluated (ALSFRS-R and rate of progression) did not reach statistical significance. The patterns of microstructural alteration observed in the white matter tracts analyzed showed a spatial distribution consistent with the typical clinical manifestations of ALS. However, the finding of greater involvement in the left hemisphere in our study population did not correlate with the laterality of the onset of motor symptoms reported by the patients.

## 4 Discussion

Our findings provide several insights into ALS pathophysiology. First, the asymmetric nature of white matter changes suggests that disease progression may not be uniform across hemispheres. Second, the involvement of non-motor pathways supports the contemporary view of ALS as a complex neurodegenerative disorder affecting multiple neural systems.

This study employed a dual analytical approach to assess white matter alterations in ALS patients in a comprehensive manner. The combination of whole-brain voxelwise analysis and tract-specific examination allowed for a nuanced understanding of white matter integrity.

DKI analysis in ALS patients revealed significant white matter alterations compared to healthy controls. In neurodegenerative diseases, overall white matter microstructural damage is typically expressed by increased MD and decreased FA, whereas RD and AD are more specific markers of myelin and axon degeneration, respectively. Although our study reproduced most of the expected results, it found a paradoxical increase in AD, suggesting a more complex pattern of neurodegeneration.

The comprehensive pattern of involvement across multiple diffusion metrics corroborates our tract-specific findings and provides further evidence of asymmetric motor pathway involvement in ALS. Left gray and white matter asymmetry has been previously described in volumetric and DTI studies and is postulated to represent an increased vulnerability in the dominant motor cortex in right-handed patients, regardless of the laterality of symptoms at disease onset (Devine et al., 2015; Menke et al., 2012).

DKI analysis revealed significant white matter alterations, with prominent changes in the CST and additional involvement of the FPT and PPT tracts. The evidence, obtained by tract-specific and whole-brain analyzes, demonstrates that white matter degeneration extends beyond primary motor pathways, especially involving sensorimotor integration regions (TPF segments 60–80) and suggesting a pattern of disease spread along functionally connected pathways.

Regarding the lack of statistical significance in the segments proximal to the motor cortex observed in Figure 3, this phenomenon can be explained by inherent limitations of tractography reconstruction. The variability in the termination of the reconstructed streamlines represents a known technical challenge: some streamlines terminate prematurely due to limitations in the tractography algorithm when faced with areas of low anisotropy or fiber crossings, while others reach the cortex with greater extension. This heterogeneity in the reconstruction generates greater statistical variability in the diffusion values projected precisely in these cortical segments, reducing the statistical power to detect differences between groups. This phenomenon has been documented in previous tractography studies (Garyfallidis et al., 2012) and represents a methodological limitation rather than a biological finding in itself.

The findings, validated by both tract-specific (BUAN) and whole-brain (TBSS) analyses, highlight ALS as an integrative neural network disorder affecting motor planning and execution. Three-dimensional reconstructions confirm this spatial distribution of changes, which follows a pattern parallel to that observed in the corticospinal tract, providing evidence that ALS pathology impacts networks beyond primary motor pathways and suggesting broader implications for understanding the full spectrum of the disease.

While our study establishes that DKI is sensitive to ALS-related white matter pathology based on previous investigations demostrating its superior performance compared to DTI (Zhu et al., 2015; Huang et al., 2020), certain limitations must be acknowledged. The limited sample size prevents consideration of the substantial heterogeneity of ALS, both in terms of phenotype and prognosis. Future research directions should focus on multicenter cohorts to standardize protocols and expand subtype-specific analyses. Combining DKI with other biomarkers could further elucidate structure-function relationships in ALS, potentially refining its role in therapeutic trials and personalized prognostic models.

## Data Availability

The data analyzed in this study is subject to the following licenses/restrictions: the dataset contains anonymized hospital neuroimaging data. Access is restricted by European patient privacy regulations. All participants provided written informed consent. Data requests should be directed to the corresponding author. Requests to access these datasets should be directed to Juan Quizhpilema, juan.quizhpilema@unavarra.es.
